# Ganoderic Acid A Inhibits High Glucose-Induced Oxidative Stress and Extracellular Matrix Accumulation in Rat Glomerular Mesangial Cells

This article has been retracted.

**DOI:** 10.1155/2022/5249910

**Published:** 2022-10-13

**Authors:** Jing Wang, Bing Wu, Yanting Zhu, Gang Jin, Xiaobao Fan

**Affiliations:** Center of Kidney Dialysis, The Shaanxi Provincial People's Hospital, Xi'an 710068, China

## Abstract

**Objective:**

We aimed to investigate the role of ganoderic acid A (GAA) in glomerular mesangial cells (GMCs) under high glucose (HG).

**Methods:**

GMCs were pretreated with GAA and then cultured under HG condition for 24 h. Cell proliferation was measured by CCK-8 assay. The production of intracellular ROS was determined using DCFH-DA. The activities of SOD and CAT were measured using ELISA kits. The expressions of NOX2, NOX4, fibronectin (FN), collagen IV (col IV), p38, and p-p38 were detected by western blot.

**Results:**

GAA suppressed GMC proliferation in response to HG stimulation. GAA significantly attenuated HG-caused increase in ROS production and decreases in SOD and CAT activities in GMCs. In addition, the increased expressions of NOX2 and NOX4 and NOX activity in HG-induced GMCs were significantly decreased by GAA. Furthermore, GAA greatly inhibited the levels of FN and col IV in HG-stimulated GMCs. Mechanistic investigations showed that HG caused activation of p38 MAPK pathway, whereas the induction was mitigated by GAA. Notably, the specific agonist of p38 MAPK pathway (P79350) reversed the effects of GAA on GMCs.

**Conclusion:**

GAA protected GMCs from HG-induced oxidative stress and ECM production, which was mediated by the inhibition of the p38 MAPK pathway.

## 1. Introduction

Diabetic nephropathy (DN) is a major complication of diabetes and supervenes as the result of microvascular lesions in the renal glomeruli [1, 2]. DN is characterized by glomerular hypertrophy, proteinuria, and renal fibrosis, which finally result in the loss of renal function [3]. The occurrence of DN is associated with factors such as advanced age, long course of disease, hyperglycemia, hypertension, obesity, hyperlipidemia, and high-sodium diet. Clinical studies have shown that DN accounts for about 10%-40% of patients with type 2 diabetes in China. Due to the insidious early clinical symptoms of DN, the disease has progressed to the middle and late stage, and the disease is irreversible once the typical symptoms such as edema, polyuria or oliguria, or even urinary retention occur. Therefore, early diagnosis and early comprehensive treatment of DN are especially important. At present, there is no effective western medicine to treat DN. The basic comprehensive treatment for DN involves lifestyle intervention (such as exercise, weight loss, smoking cessation, and salt restriction), control of blood sugar and blood pressure, and correction of metabolic disorders. Currently, there are clinical studies showing that traditional Chinese medicine for nourishing qi, nourishing yin, promoting blood circulation, and removing blood stasis can play a positive role in the prevention of DN.

Additionally, patients with DN have very high cardiovascular risk [1, 4]. Therefore, timely diagnosis and effective management of DN are of paramount importance. Numerous efforts have been made to explore molecular mechanisms in the pathogenesis of this disease. Several mechanisms have been postulated to be closely related with DN progression, such as hyperglycemia, increased oxidative stress, and production of cytokines and chemokines [5]. Among these mechanistic insights, oxidative stress plays a critical role in propagation of DN [6, 7]. The increased oxidative stress causes activation of inflammatory and apoptotic signals, which leads to renal injury in the pathogenesis of DN [3, 8]. Many evidences suggest the importance of glomerular mesangial cells (GMCs) in the progression of DN [9]. In addition to oxidative damage, hyperglycemia also promotes cell proliferation and extracellular matrix (ECM) synthesis in GMCs, thereby contributing to glomerular hypertrophy and fibrotic events. Hyperglycemia can mediate kidney damage in diabetes through a variety of molecular mechanisms, including oxidative stress, proinflammatory cytokines, induction of transforming growth factor-*β*1 expression, activation of fibroblasts, and the renin-angiotensin system. Hence, it is urgent to find new agent protecting GMCs from hyperglycemia.

In the field of traditional Chinese medicine in China, Ganoderma lucidum has been recognized as a promising remedy. “Compendium of Materia Medica” records: “Ganoderma lucidum is flat, bitter in taste, non-toxic, and can invigorate the heart, nourish the middle, and enhance wisdom.” Modern medicine has also researched and explored the pharmacological effects of Ganoderma lucidum and found that it has the functions of immune regulation, liver protection, antitumor, and treatment of cardiovascular diseases. Ganoderic acid A (GAA) is the major triterpenoid component extracted from *Ganoderma lucidum*. Many publications have demonstrated that GAA has broad biological activities, such as antioxidative, antibacterial, and anti-inflammatory [10–12]. Notably, GAA was found to have the capacity for the treatment of diabetic complications. Zhu et al. reported that GAA improves insulin sensitivity in high-fat diet- (HFD-) induced obese mice [13]. However, the role of GAA in DN is still unclear.

## 2. Materials and Methods

The study protocol and all amendments were approved by the appropriate ethics committee at each center (NI-WU20200102). The study was done in accordance with the protocol, its amendments, and standards of Clinical Practice. All participants provided written informed consent before enrolment.

### 2.1. Cell Culture

Rat GMCs line (HBZY-1 cells) was obtained from ATCC and cultured in RPMI-1640 medium supplemented with 10% FBS at 37°C. Cells were grown under normal glucose condition (5.5 mM glucose) or high glucose condition (30 mM glucose).

### 2.2. Cell Cytotoxicity Assay

Cell cytotoxicity was tested by MTT assay after incubating with different concentrations of GAA (0-40 *μ*g/ml) for 24 h. After the treatment, 100 *μ*l of MTT solution (5 mg/ml) was added to each well. The formazan crystals were solubilized in DMSO. The OD value was read on a microplate reader.

### 2.3. Cell Proliferation Assay

Briefly, cells (5 × 10^3^ cells/well) were plated and cultured with different concentrations of GAA (5, 10, and 20 *μ*g/ml) under NG condition (5.5 mM) or HG condition (30 mM). After incubation for 24 h, cells were added with CCK-8 solution and incubated for 4 h. The absorbance (450 nm) was measured using a microplate reader.

### 2.4. Intracellular ROS Measurement

The production of intracellular ROS was determined using an oxidant-sensitive probe DCFH-DA. The treated HBZY-1 cells were incubated with DCFH-DA for 30 min in the dark. The fluorescence intensity was detected by fluorescence spectrophotometer with an excitation wavelength of 502 nm and an emission wavelength of 523 nm.

### 2.5. Activities of SOD and CAT

After treatment, the supernatant was collected for the determination of SOD and CAT activities by commercial kits.

### 2.6. NOX Activity Detection

NOX activity in cell lysates was measured by chemiluminescence method using a commercial assay kit. Then, the NOX activity was determined at 340 nm using spectrophotometry (Thermo Scientific, Rockford, IL, USA).

### 2.7. Detection of FN and col IV

After different treatments, cell culture medium was harvested and centrifuged. Then, the supernatants were collected for detecting FN and collagen IV production using commercial ELISA kits.

### 2.8. Western Blot

Cell lysates were run on 10% SDS-PAGE and electrotransferred to nitrocellulose membranes. Then, the membranes were blocked, followed by incubating with rabbit anti-rat monoclonal antibodies against NOX2, NOX4, FN, col IV, p38 MAP kinase (p38 MAPK), p-p38, and *β*-actin (Abcam). After overnight incubation at 4°C, the membranes were incubated with HRP-conjugated secondary antibody. The immunoreactive protein complex was detected by ECL kit.

### 2.9. Statistical Analysis

The normality of the sample was determined with the Shapiro–Wilk test. Descriptive statistical data were evaluated with the exploratory analyses of the Tukey test. Quantitative mean data (PES/WES, ISQ, and B.L.) were assessed with the nonparametric Wilcoxon-Mann–Whitney *U* test to analyze the inferential statistical. Data were presented as means ± SEM. Differences among different groups were assessed by ANOVA followed by Tukey post hoc test. *p* < 0.05 was considered statistically significant.

## 3. Results

### 3.1. GAA Suppresses GMC Proliferation

To evaluate the cytotoxicity effect of GAA on GMCs, we adopted the MTT assay. The concentrations of GAA (5, 10, and 20 *μ*g/ml) treatment did not affect GMC viability (Figure 1(a)). The concentrations of 5-20 *μ*g/ml were used for the further investigations. Then, we explored the effect of GAA on GMC proliferation in response to HG stimulation. As indicated in Figure 1(b), HG stimulation significantly promoted GMC proliferation; however, GAA treatment suppressed HG-promoted MC proliferation.

### 3.2. GAA Inhibits Oxidative Stress in GMCs

To assess the importance of GAA in oxidative stress, we detected ROS production in GMCs. In Figure 2(a), ROS production was increased in HG-stimulated GMCs, compared with control GMCs. The elevated ROS production was reduced by GAA pretreatment. Also, the decreased activities of SOD and CAT caused by HG stimulation were also attenuated by GAA pretreatment (Figures 2(b) and 2(c)).

### 3.3. GAA Inhibits the Expressions of NOX2/4 in HG-Stimulated GMCs

NOX2 and NOX4 are two major subtypes of NOX that are important for the generation of ROS. The protein expressions of NOX2 and NOX4 were, respectively, increased by HG. However, the increased NOX2 and NOX4 expressions were decreased in GAA pretreated cells (Figures 3(a)–3(c)). Additionally, GAA reduced HG-mediated increase in NOX activity in GMCs (Figure 3(d)).

### 3.4. GAA Inhibits ECM Accumulation in GMCs

Next, the effect of GAA on FN and col IV production was measured. ELISA proved that the levels of FN and col IV in the culture supernatant were markedly increased by HG. After pretreated with GAA, FN and col IV contents were decreased (Figures 4(a) and 4(b)). Furthermore, the expressions of two proteins in GMCs were determined. As illustrated in Figures 4(c) and 4(d), HG markedly stimulated the expressions of two proteins in GMCs, while these effects were mitigated by GAA.

### 3.5. GAA Inhibits p38 MAPK Pathway Activation in GMCs

The p38 MAPK pathway plays a crucial role in GMCs in response to the HG stimulation. Then, we further tested the effect of GAA on this pathway. HG stimulation caused an obvious increase in p-p38 expression in GMCs, whereas treatment with GAA significantly reduced the phosphorylation of p38 (Figure 5).

### 3.6. P79350 Reversed the Effect of GAA on Oxidative Stress in GMCs

To further confirm the role of the p38 MAPK pathway, GMCs were incubated with P79350 (10 nM), a specific agonist of the p38 MAPK pathway. As indicated in Figures 6(a) and 6(b), P79350 significantly increased the level of p-p38 in GMCs treated with GAA following HG stimulation. In addition, the decreased cell proliferation and ROS production, as well the increased activities of SOD and CAT in GAA-treated cells were dramatically attenuated by P79350 (Figures 6(c)–6(f)).

### 3.7. P79350 Reversed the Effect of GAA on ECM

Furthermore, the effect of P79350 on GAA-regulated ECM accumulation in GMCs exposed to HG was investigated. The data demonstrated that the inhibitory effect of GAA on FN and col IV production was significantly reversed by P79350 in HG-treated GMCs (Figures 7(a) and 7(b)).

## 4. Discussion

Diabetes is a chronic metabolic disease, and it has high plasma glucose level. It is well known that prolonged exposure to high glucose levels results in mitochondrial overproduction of ROS [14]. The imbalance between increased intracellular ROS and their neutralization results in oxidative stress, which is considered as the most important event [15]. Accumulation of ROS and ROS-mediated oxidative stress can trigger a number of abnormal pathways. Subsequently, it may increase mesangial expansion and glomerulosclerosis [6, 14]. Therefore, scavenging ROS under HG condition may be useful for attenuating DN. DN is one of the most common microvascular complications of diabetes and the main cause of end-stage renal disease and chronic kidney disease. The main clinical feature is persistent albuminuria and/or progressive decline in glomerular rate filtration (GFR) and can develop into end-stage renal disease. In the early stage of DN, abnormal renal function, proteinuria, edema, and anemia may occur. A large amount of proteinuria may gradually produce with the absence of timely intervention. In severe cases, it may develop into uremia and endanger the life safety of patients. Therefore, early blood sugar control is required to protect renal function, reduce proteinuria, and prevent further deterioration of the condition.

Proliferation of GMCs is an important event that contributes to DN progress. We found that GAA suppressed the cell proliferation of GMCs in response to HG stimulation. In addition, GAA attenuated HG-caused increase in ROS production and decrease in SOD and CAT activities, indicating that GAA mitigated HG-induced oxidative stress. In the diabetic kidney, NOX is the main source of ROS and thereby promotes pathophysiological events in kidney disease [14, 16]. Our data showed that GAA reduced the expressions of NOX2 and NOX4, which might contribute to the inhibition of ROS production. It has been demonstrated that increased ROS production can activate various signaling pathways, therefore promoting the progression of mesangial expansion and glomerulosclerosis [17, 18].

In the present study, we revealed that the expressions of FN and col IV were decreased by GAA treatment. Collectively, GAA suppressed cell proliferation, ROS production, and ECM accumulation in GMCs, indicating GAA might have potential role in attenuating DN. The activation of inflammatory and apoptosis induced by oxidative stress are two major events in the development of DN [19]. Oxidative stress can cause glomerulosclerosis through various pathogenic mechanisms such as inflammation, fibrosis, and metabolic disorders and also damage the physiological function and structure of renal tubules, aggravating the process of DN. Glucose itself can induce oxidative stress, and the advanced glycation end products (AGEs) produced in the metabolic process can also aggravate the oxidative stress of HMC, causing glomerulosclerosis and renal tubular inflammation, fibrosis, and apoptosis, and ultimately lead to the occurrence and development of DN.

Among various signaling pathways, MAPKs are considered one of the main mechanisms mediated by ROS [5, 20, 21]. MAPKs are critical components for the extracellular stimulus-mediated signal transduction process including ERK, JNK, and p38 MAPK [22]. Activation of p38 MAPK is related with renal injury. In addition, p38 activity is increased in glomeruli and mesangial cells during the development of DN. Exposure to HG condition also activates p38 MAPK in human mesangial cells [23–25]. Previous results have suggested that suppression of p38 MAPK is lethal for DN patients. Our results proved that the p38 MAPK was activated in response to HG condition, whereas GAA repressed p38 MAPK activation. Treatment with the specific agonist of this pathway abolished the effects of GAA on HG-induced GMCs. These results denoted that GAA executed its roles via inhibiting the p38 MAPK pathway. In addition, mesangial cells are an important part of maintaining the normal shape and function of the glomerulus, and their main role is to maintain the integrity of the glomerular capillary network. Cultivating MES-13 cells in high-glucose medium will increase the content of intracellular ROS and lead to the occurrence of apoptosis.

Our findings demonstrate that ganoderic Acid A inhibits high glucose-induced oxidative stress and extracellular matrix accumulation in rat glomerular mesangial cells, which provides some ideas for future DN treatment. This study not only proves once again that the pathogenesis of DN is related to oxidative stress but also provides new research findings for traditional Chinese medicine treatment. However, future in vitro and in vivo experiments are required to validate our results.

In conclusion, GAA has a protective effect on HG-induced GMCs with deceased ROS production, oxidative stress, and ECM accumulation. The possible mechanism was associated with inhibition of p38 MAPK pathway. The results suggested that GAA might be an alternative choice for the prevention and management of DN. However, further studies are required to illuminate the biological activities of GAA in an *in vivo* DN model.

## Figures and Tables

**Figure 1:** GAA alleviates HG-induced cell proliferation of GMCs. (a) Following incubation with different concentrations of GAA (0, 5, 10, 20, and 40 *μ*g/ml) for 24 h, cell cytotoxicity was evaluated by MTT assay. ^∗^*p* < 0.05 vs. the control group. (b) GMCs were pretreated with 5, 10, and 20 *μ*g/ml of GAA and then cultured under NG or HG condition for 24 h; then, cell proliferation was measured by CCK-8 assay. ^∗^*p* < 0.05 vs. the NG group, ^#^*p* < 0.05 vs. the HG group.

**Figure 2:** GAA inhibits HG-stimulated oxidative stress in GMCs. GMCs were pretreated with 5, 10, and 20 *μ*g/ml of GAA and then cultured under NG or HG condition for 24 h. (a) Effect of GAA on ROS production. (b, c) Effects of GAA on activities of SOD and CAT. ^∗^*p* < 0.05 vs. the NG group, ^#^*p* < 0.05 vs. the HG group.

**Figure 3:** GAA inhibits the HG-stimulated expressions of NOX2/4 and NOX activity in GMCs. GMCs were pretreated with 5, 10, and 20 *μ*g/ml of GAA, followed by an incubation under NG or HG condition for 24 h. (a) The expressions of NOX2 and NOX4 were detected by western blot analysis. (b, c) Quantification analysis of NOX2 and NOX4. (d) Effect of PSP on NOX activity. ^∗^*p* < 0.05 vs. the NG group, ^#^*p* < 0.05 vs. the HG group.

**Figure 4:** GAA inhibits HG-stimulated ECM accumulation in GMCs. GMCs were pretreated with 5, 10, and 20 *μ*g/ml of GAA, followed by an incubation under NG or HG condition for 24 h. (a, b) The levels of FN and col IV in culture supernatant were detected using ELISA. (c) The expressions of FN and col IV in GMCs were detected by western blot analysis. (d) Quantification analysis of FN and col IV. ^∗^*p* < 0.05 vs. the NG group, ^#^*p* < 0.05 vs. the HG group.

**Figure 5:** GAA inhibits the HG-stimulated activation of p38 MAPK pathway in GMCs. GMCs were pretreated with 5, 10, and 20 *μ*g/ml of GAA, followed by an incubation under NG or HG condition for 24 h. (a) The expression levels of p38 and p-p38 were detected by western blot analysis. (b) Quantification analysis of p-p38/p38. ^∗^*p* < 0.05 vs. the NG group, ^#^*p* < 0.05 vs. the HG group.

**Figure 6:** Activation of p38 MAPK reversed the protective effect of GAA on oxidative stress in HG-stimulated GMCs. GMCs were incubated with P79350 (10 nM) and/or GAA (20 *μ*g/ml), followed by an incubation under NG or HG condition for 24 h. (a) The expression levels of p38 and p-p38 were detected by western blot analysis. (b) The ratio of p-p38/p38. (c) Cell proliferation was measured by CCK-8 assay. (d) The production of intracellular ROS was determined using DCFH-DA. (e, f) The activities of SOD and CAT were measured using ELISA kits. ^∗^*p* < 0.05 vs. the NG group, ^#^*p* < 0.05 vs. the HG group, and ^&^*p* < 0.05 vs. the HG+GAA group.

**Figure 7:** Activation of p38 MAPK reversed the protective effect of GAA on ECM production in HG-stimulated GMCs. GMCs were incubated with P79350 (10 nM) and/or GAA (20 *μ*g/ml), followed by an incubation under NG or HG condition for 24 h. (a, b) The productions of FN and col IV were detected using ELISA kits. ^∗^*p* < 0.05 vs. the NG group, ^#^*p* < 0.05 vs. the HG group, and ^&^*p* < 0.05 vs. the HG+GAA group.

## Data Availability

Data are available upon reasonable request. The data that support the findings in this study are available from the corresponding author upon request.
